# Influence of *DPYD* Genetic Polymorphisms on 5-Fluorouracil Toxicities in Patients with Colorectal Cancer: A Meta-Analysis

**DOI:** 10.1155/2014/827989

**Published:** 2014-12-28

**Authors:** Qiang Li, Ying Liu, Hong-Mei Zhang, Yin-Peng Huang, Tian-Yi Wang, Dong-Sheng Li, Hong-Zhi Sun

**Affiliations:** ^1^Department of Oncology, Jining No. 1 People's Hospital, No. 6 Jiankang Road, Jining, Shandong 272011, China; ^2^Department of Immunology, Laiwu Municipal Center for Disease Control & Prevention, Laiwu 271100, China

## Abstract

Our meta-analysis aggregated existing results from relevant studies to comprehensively investigate the correlations between genetic polymorphisms in dihydropyrimidine dehydrogenase (*DPYD*) gene and 5-fluorouracil (5-FU) toxicities in patients with colorectal cancer (CRC). The MEDLINE (1966∼2013), the Cochrane Library Database (Issue 12, 2013), EMBASE (1980∼2013), CINAHL (1982∼2013), Web of Science (1945∼2013), and the Chinese Biomedical Database (CBM) (1982∼2013) were searched without language restrictions. Meta-analyses were conducted with the use of STATA software (Version 12.0, Stata Corporation, College Station, TX, USA). Seven clinical cohort studies with a total of 946 CRC patients met our inclusion criteria, and NOS scores of each of the included studies were ≥5. Our findings showed that *DPYD* genetic polymorphisms were significantly correlated with high incidences of 5-FU-related toxicity in CRC patients. SNP-stratified analysis indicated that there were remarkable connections of IVS14+1G>A, 464T>A, and 2194G>A polymorphisms with the incidence of marrow suppression in CRC patients receiving 5-FU chemotherapy. Furthermore, we found that IVS14+1G>A, 496A>G, and 2194G>A polymorphisms were correlated with the incidence of gastrointestinal reaction. Ethnicity-stratified analysis also revealed that *DPYD* genetic polymorphisms might contribute to the development of marrow suppression and gastrointestinal reaction among Asians, but not among Caucasians. The present meta-analysis suggests that *DPYD* genetic polymorphisms may be correlated with the incidence of 5-FU-related toxicity in CRC patients.

## 1. Introduction

Colorectal cancer (CRC) is a malignant tumor caused by uncontrolled cell growth in the colon or rectum, or in the appendix, which is typically manifested by rectal bleeding, anemia, weight loss, and changes in bowel habits [1]. According to the statistics, CRC is the most common malignant cancer expected to occur in both men and women, as well as the most common cause of cancer death in 2013 [2]. Generally, CRC is considered to be a heterogeneous group of complex diseases, and surgical resection and chemotherapy have widely been used in the treatment of CRC patients during the past decades [3, 4]. Recently, many studies showed that adjuvant chemotherapy with 5-fluorouracil (5-FU), which is a pyrimidine analog drug used in the treatment of cancer, could be an effective strategy for CRC treatment [5, 6]. However, several clinical reports have shown that some factors, including the activity of dihydropyrimidine dehydrogenase (DPYD) which was responsible for drug catabolism, may contribute to interpatient variability of 5-FU pharmacokinetics [7, 8]. Recently, extensive studies have suggested that single nucleotide polymorphism (SNP) may be associated with toxicity of 5-FU adjuvant chemotherapy in CRC [9, 10].

DPYD, acting as a pyrimidine catabolic enzyme, is suggested to be the initial and rate-limiting factor in the catabolism pathway of 5-FU toxic metabolites [11]. It has been well established that the deficiency of DPYD is closely linked to the 5-FU-related toxicities, such as stomatitis, mucositis, diarrhea, and neurotoxicity [12]. Indeed, activity of proteins related to the pharmacokinetics and pharmacodynamics of 5-FU may explain the intolerance in CRC patients [13]. Particularly, the DPD enzyme encoded by the* DPYD* gene has been identified to play a crucial role in the pharmacology of 5-FU in CRC patients receiving chemotherapy [14]. Consequently, understanding of the relationship of DPYD and pharmacology of 5-FU may lead to decreased incidence of adverse drug events and possible improved survival of CRC patients [11, 13]. Human* DPYD* gene is located on chromosome 1p22, encompassing 23 exons and spanning approximately 843 kb [15]. Genetic polymorphisms in the* DPYD* gene may contribute to decreased activations of DPD enzyme which result in reduced clearance of 5-FU and thereby conduce to increased toxicity of 5-FU in CRC patients [16]. In recent years, several SNP, including IVS14+1G>A, 464T>A, 2194G>A, 496A>G, and 1627A>G, in the* DPYD* gene have been investigated to be related to toxicity of 5-FU chemotherapy in CRC patients [13, 14, 16]. The most frequently described genetic variant of the* DPYD* gene in CRC patients with partial or complete DPD deficiency is a G to A point mutation within the 5′-splicing donor site of intron 14 [9]. Furthermore, a large number of human studies have supported the fact that* DPYD* genetic polymorphisms are potentially useful markers of the response to 5-FU chemotherapy [9, 11], but contradictory results were also reported [17, 18]. Therefore, we conducted this update meta-analysis to explore whether genetic polymorphisms in the* DPYD* gene are correlated with 5-FU-related toxicity in CRC patients.

## 2. Methods

### 2.1. Literature Search and Selection Criteria

The MEDLINE (1966~2013), the Cochrane Library Database (Issue 12, 2013), EMBASE (1980~2013), CINAHL (1982~2013), Web of Science (1945~2013), and the Chinese Biomedical Database (CBM) (1982~2013) were searched without language restrictions. We used the following keywords and MeSH terms in conjunction with a highly sensitive search strategy: (“genetic polymorphism” or “single nucleotide polymorphism” or “polymorphism“ or “SNP” or “mutation” or “variation” or “variant”) and (“dihydrouracils dehydrogenase” or “NADP” or “DPYD” or “DPD”) and (“colorectal cancer” or “colorectal carcinogenesis” or “colorectal tumor” or “colorectal carcinoma” or “large intestine cancer” or “large intestine carcinoma” or “large colon cancer” or “large bowel cancer”). A manual search on the basis of references identified in the included articles was performed to obtain other potential articles.

The following criteria were utilized to identify the eligibility of included studies: (1) the study must concern the correlations between* DPYD* genetic polymorphisms and toxicity of 5-FU in CRC patients; (2) all patients involved in the meta-analysis received 5-FU chemotherapy regimen for the first time, and they did not develop chronic liver disease or any liver dysfunction that may have an impact on the metabolism of 5-FU; (3) sufficient information about the frequency of* DPYD* genetic polymorphisms should be provided in the article. The articles that were not in accordance with our inclusion criteria must be excluded. If authors published several studies of the same subjects, either the most recent or the largest sample size publication was included.

### 2.2. Data Extraction and Methodological Assessment

Two authors from each included study systematically collected relevant data by using a standardized form. The most relevant items were documented in the form for data extraction, including language of publication, publication year of article, the first author's surname, geographical location, design of study, total number of cases, sample size, the source of the subjects, type of sample, detection method of genotypes, the frequency of genetic polymorphisms, gastrointestinal reaction, and adverse drug reaction.

Methodological quality was evaluated separately by two observers using the Newcastle-Ottawa Scale (NOS) criteria [19]. The NOS criteria were based on 3 aspects: (1) subject selection: 0~4; (2) comparability of subject: 0~2; (3) clinical outcome: 0~3. Total NOS scores ranged from 0 to 9 with a score ≥7 meaning a good quality.

### 2.3. Statistical Analysis

The STATA statistical software (Version 12.0, Stata Corporation, College Station, TX, USA) was employed in the meta-analysis to achieve rigorous statistical analysis. Odds ratios (OR) with their corresponding 95% confidence interval (95% CI) were calculated. The *Z* test was used to estimate the statistical significance of pooled ORs. Between-study heterogeneity was assessed by Cochran's* Q*-statistic and *I* ^2^ tests [20]. If the* Q*-test exhibited a *P* < 0.05 or the *I* ^2^ test showed >50%, which means that these studies were heterogeneous, the random-effect model was conducted; otherwise, the fixed-effects model was used. We also make use of subgroup analyses to explore sources of heterogeneity. In order to evaluate the influence of single studies on the overall estimate, a sensitivity analysis was performed. Potential publication bias was investigated with the use of Funnel plots and Egger's linear regression test [21].

## 3. Results

### 3.1. Study Selection and Characteristics of Included Studies

Initially, our highly sensitive search strategy identified 145 articles. We reviewed the titles and abstracts of all articles and excluded 68 articles; then we systematically reviewed full texts and 66 articles were further excluded. Another 4 studies were also excluded due to lack of data integrity (Figure 1). Finally, 7 clinical cohort studies with a total of 946 CRC patients met our inclusion criteria for quantitative data analysis [9, 11, 13, 17, 18, 22, 23]. The range of publication years of the eligible studies was from 2001 to 2013. Distribution of the number of topic-related literatures in the electronic database during the last decade was shown in Figure 2. Overall, 3 studies were conducted among Caucasians and another 4 studies among Asians. Seven common polymorphisms in the* DPYD* gene were assessed, including IVS14+1G>A, 85T>C, 464T>A, 2194G>A, 496A>G, 1896T>C, and 1627A>G. None of the studies deviated from the HWE (all *P* < 0.05). NOS scores of each of the included studies were ≥5. The characteristics and methodological quality of included studies were collected in Table 1.

### 3.2. Quantitative Data Synthesis

Meta-analysis results showed that patients with* DPYD* genetic polymorphisms had a higher incidence of marrow suppression than those without* DPYD* genetic variants (OR = 6.81, 95% CI: 2.85~16.29, *P* < 0.001). Furthermore, we observed that there were significant correlations between* DPYD* genetic polymorphisms and the occurrence of gastrointestinal reaction (OR = 1.93, 95% CI: 1.20~3.10, *P* = 0.007) and hand-foot syndrome (OR = 1.22, 95% CI: 1.00~1.48, *P* = 0.048) in CRC patients (Figure 3).

In SNP-stratified subgroup, our results indicated that there were remarkable connections of IVS14+1G>A, 464T>A, and 2194G>A polymorphisms with the incidence of marrow suppression in CRC patients receiving 5-FU chemotherapy (all *P* < 0.05) (Figure 4). However, we found no associations of 85T>C, 496A>G, 1896T>C, or 1627A>G with the incidence of marrow suppression (all *P* > 0.05). Furthermore, we found that IVS14+1G>A, 496A>G, and 2194G>A polymorphisms were correlated with the occurrence of gastrointestinal reaction (all *P* < 0.05), but similar correlations were not found in other polymorphisms (all *P* > 0.05). Among different ethnicities, the findings revealed that* DPYD* genetic polymorphisms might contribute to the development of marrow suppression and gastrointestinal reaction among Asians (marrow suppression: OR = 12.05, 95% CI: 3.94~36.85, *P* < 0.001; gastrointestinal reaction: OR = 4.39, 95% CI: 2.75~6.99, *P* < 0.001, resp.), but no similar results were found among Caucasians (all *P* > 0.05) (Figure 4). Moreover, the results of subgroup analysis by sample size showed significant relationships of* DPYD* genetic polymorphisms with marrow suppression and gastrointestinal reaction in CRC patients in the majority of subgroups.

A sensitivity analysis was performed to assess the influence of each individual study on the pooled estimates by omitting individual studies. The outcomes suggested that no single study could influence the pooled ORs (Figure 5). Funnel plots demonstrated no evidence of obvious asymmetry existing (Figure 6). No publication bias was found by Egger's test (all *P* > 0.05).

## 4. Discussion

In the current meta-analysis, we evaluated the relationships between* DPYD* genetic polymorphisms and toxicity of 5-FU in CRC patients. The results of our meta-analysis showed significant correlations between* DPYD* genetic polymorphisms and the incidence of adverse drug events in CRC patients receiving 5-FU chemotherapy, including marrow suppression, gastrointestinal reaction, and hand-foot syndrome, implying that* DPYD* genetic polymorphisms may be significantly related to toxicity of 5-FU chemotherapy in CRC. Nevertheless, the precise mechanism by which* DPYD* genetic polymorphisms lead to enhanced toxicity of 5-FU in CRC patients is still largely unknown. It is well established that 5-FU is an important component of many standard treatments in the multimodal therapy of CRC, which always induces side effects and toxicity-related death unfortunately [9]. It should be noted that DPYD acts as a rate-limiting enzyme in the catabolism of 5-FU, converting 5-FU to 5-fluorodihydrouracil (FDHU), which is further metabolized to its final metabolite 5-fluoro-b-alanine excreted in the urine [16]. In particular, the deficiency of DPYD enzyme activity is closely related to a delay in the clearance of 5-FU, which may inevitably enhance the toxic side effects of 5-FU [23]. We therefore hypothesized that* DPYD* genetic polymorphisms might alter the expression and function of DPYD and may decrease its ability in clearance of 5-FU [11]. Thus, it was plausible that* DPYD* genetic polymorphisms may contribute to reinforced 5-FU toxicity. The findings are in accordance with a previous study which demonstrated an allele-dose dependent association of the nonsynonymous sequence aberration c.496A>G and indicated that the methionine-valine exchange caused by the c.496A>G transition has posed a deleterious effect on DPYD deficient patients [14]. Moreover, Kristensen et al. also revealed that sequence variations in the* DPYD* gene may influence the breakdown of the common anticancer drug 5-FU and provoke severe drug adverse effects in CRC patients receiving 5-FU therapy [9].

To investigate the influence of potential factors on the specific marrow suppression and gastrointestinal reaction of CRC patients receiving 5-FU chemotherapy, we carried out stratified analysis based on SNP and ethnicity. In the subgroup stratified by SNP, our results indicated that there was a significant association of IVS14+1G>A, 464T>A, and 2194G>A polymorphisms with the incidence of marrow suppression in CRC patients receiving 5-FU chemotherapy. In addition, we found that IVS14+1G>A, 496A>G, and 2194G>A polymorphisms were associated with the occurrence of gastrointestinal reaction. Among different ethnicities,* DPYD* genetic polymorphisms showed a close relationship with the development of marrow suppression and gastrointestinal reaction in Asians, revealing that there was ethnic difference in the effects of* DPYD* genetic polymorphisms on clinical outcome of 5-FU chemotherapy. Although the potential mechanism of ethnicity differences is still not fully understood, we supposed that ethnicity may result in differences in alleles and genotypes among different ethnic populations.

Our meta-analysis also has a number of potential limitations. Firstly, due to the small number of studies, our results did not include all the data from all trials to assess the correlations between* DPYD* genetic polymorphisms and toxicity of 5-FU in CRC patients, which may have a negative effect on the general applicability of our findings. Consequently, the cognitive function of our meta-analysis should be considered elementary. A second limitation of our meta-analysis is the fact that, as a retrospective study, there are no guidelines as to how much information a meta-analysis should include to be reliable, which may explain why many controversies occur when the results of meta-analysis and large trials were not consistent. Another potential limitation is that our meta-analysis was unable to acquire original data from the included studies. Even though our meta-analysis has the above limitations, this is the first meta-analysis on the association between* DPYD* genetic polymorphisms and toxicity of 5-FU in CRC patients. More importantly, our meta-analysis has a clear selection criterion in literature search strategy. In order to achieve strong objectivity, all the research methods were based on strict inclusion and exclusion criteria. Besides, meta-analysis undertaken according to these rigorous statistical analyses will lead to a more reliable conclusion.

## 5. Conclusions

To sum up, the present meta-analysis suggested that* DPYD* genetic polymorphisms might be correlated with the incidence of marrow suppression, gastrointestinal reaction, and hand-foot syndrome. Therefore,* DPYD* genetic polymorphisms may be valuable in predicting toxicity of 5-FU in CRC patients. However, for the fact that several limitations existed in our meta-analysis, larger sample size studies with more integral data are needed to obtain a more profound and representative statistical analysis.

## Figures and Tables

**Figure 1:** Flow chart showing study selection procedure. Seven cohort studies were included in this meta-analysis.

**Figure 2:** The distribution of the number of topic-related literatures in electronic databases over the last decade.

**Figure 3:** Forest plots for the relationships of* DPYD* genetic polymorphisms with marrow suppression, gastrointestinal reaction, and hand-foot syndrome in colorectal cancer patients.

**Figure 4:** Subgroup analyses based SNP, ethnicity, and sample size for the relationships of* DPYD* genetic polymorphisms with marrow suppression and gastrointestinal reaction in colorectal cancer patients.

**Figure 5:** Sensitivity analysis for the relationships of* DPYD* genetic polymorphisms with marrow suppression, gastrointestinal reaction, and hand-foot syndrome in colorectal cancer patients.

**Figure 6:** Funnel plot of publication biases on the relationship of* DPYD* genetic polymorphisms with marrow suppression, gastrointestinal reaction, and hand-foot syndrome in colorectal cancer patients.

**Table 1:** Main characteristics and methodological quality of all eligible studies.

First author	Year	Country	Ethnicity	Sample	Sample size	Gene	SNP	Clinical indicators	NOS score
Cai [18]	2013	China	Asians	168	Large	*DPYD *	IVS14+1G>A (rs3918290 G>A)	①③	6

Teh [11]	2013	Malaysia	Asians	26	Small	*DPYD *	1627A>G (rs1801159 A>G)	②	6
							1896T>C (rs17376848 T>C)		

							85T>C (rs1801265 T>C)		
							496A>G (rs2297595 A>G)		
Deenen [13]	2011	Netherlands	Caucasians	568	Large	*DPYD *	IVS14+1G>A (rs3918290 G>A)	②③	8
							2194G>A (rs1801160 G>A)		
							1627A>G (rs1801159 A>G)		

							85T>C (rs1801265 T>C)		
Zhang [17]	2011	China	Asians	60	Small	*DPYD *	464T>A (rs11695471 T>A)	①②	6
							2194G>A (rs1801160 G>A)		

							85T>C (rs1801265 T>C)		
Kristensen [9]	2010	Denmark	Caucasians	22	Small	*DPYD *	496A>G (rs2297595 A>G)	①②	5
							1896T>C (rs17376848 T>C)		

Zhang [22]	2007	China	Asians	74	Small	*DPYD *	1627A>G (rs1801159 A>G)	②	
							85T>C (rs1801265 T>C)		

Raida [23]	2001	Netherlands	Caucasians	25	Small	*DPYD *	IVS14+1G>A (rs3918290 G>A)	②	6

M: male; F: female; SNP: single-nucleotide polymorphisms; NOS: Newcastle-Ottawa Scale; DPYD: dihydropyrimidine dehydrogenase; ①: marrow suppression; ②: gastrointestinal reaction; ③: hand-foot syndrome.
